# Baseline comparative analysis and review of election forensics: Application to Ghana's 2012 and 2020 presidential elections

**DOI:** 10.1016/j.heliyon.2023.e18276

**Published:** 2023-07-18

**Authors:** Edmund F. Agyemang, Ezekiel N.N. Nortey, Richard Minkah, Kwame Asah-Asante

**Affiliations:** a Department of Statistics and Actuarial Science, College of Basic and Applied Sciences, University of Ghana, Ghana; b Department of Computer Science, Ashesi University, No.1 University Avenue, Berekuso, Accra, Eastern Region, Ghana; c Department of Political Science, College of Humanities, University of Ghana, Ghana

**Keywords:** Election forensics, Hartigans' dip test of unimodality, Benford's second order test of conformity, First-two digits, Ghana

## Abstract

Many allegations have been levelled against the electoral process of many countries across the world by most opposition leaders, especially when they lose a presidential election e.g. Ghana in 2012 and 2020. Therefore, the need to apply election forensic techniques to the certified election results data of valid votes count to statistically verify if some suspected or possible anomalies and irregularities exist in the voting pattern. This paper seeks to provide a comprehensive review of election forensics techniques and make a comparative analysis of Benford's Second-order test of conformity (using the first two digits) and Hartigans' dip test of unimodality to examine the existence of possible anomalies and irregularities in the 2012 and 2020 presidential elections held in Ghana. The findings of the two tests suggest that the electoral process produced possible anomalous data in the 2012 presidential election results (with an overall 16.67% suspected anomalies), whilst possible non-anomalous data was produced in the 2020 presidential election results (with an overall 0% suspected anomaly) of valid votes count. Therefore, the study recommends that for better statistical data analysis on election anomaly detection, Benford's test of conformity and Hartigans' dip test of unimodality should serve as baseline tests (initial screening tools), highlighting areas that may require further investigation or more rigorous analysis and progressively dig deeper into the application of finite mixture fraud models and machine learning techniques. In spite of the promising results Benford's Law, dip test, machine learning algorithms, and network analysis have produced in detecting irregularities in election data, real-world applications remain challenging, particularly when dealing with complex and evolving forms of fraud. Therefore, there is the need for continuous research and innovation to improve the accuracy and effectiveness of these methods and promote transparency and accountability in democratic societies.

## 1 Introduction

For three decades, Ghana's democracy has seen tremendous improvement. Responsible for this are several factors, including elections that have been organized since the return to democratic rule in 1992. During this period, the conduct of most of the polls has been commended by local and international observers and agencies. However, there have been grave concerns about the quality of some elections, particularly those in 1992, 2012 and 2020. Claims of irregularities, including bloated registers, vote buying and ballot stuffing, have been cited. Allegations of irregularities in the 1992 presidential election led to a boycott of the subsequent parliamentary elections by four major parties. The main opposition party, New Patriotic Party (NPP), published a book in 1992 entitled, “The Stolen Verdict”. This account chronicled all the alleged irregularities in that election [1], [2], [3], [4], [5], [6], [7]. The purpose of election forensics is to analyze and assess election integrity, specifically when there are concerns about fraud, irregularities, or other factors that could undermine its fairness. A wide range of techniques and approaches can be incorporated into this type of analysis, including statistical analysis, physical security assessment, and ballot design analysis. Ghana's 2012 and 2020 election results were challenged in the supreme court, with the plaintiff parties claiming the polls were vitiated and this makes it ideal to statistically check for possible or suspected anomaly claims. In Ghana, election anomaly detection has not been subject to attempts at using rigorous statistical methods except [8] through the applicability of digit-based analysis and [9] through the employment of a Dirichlet Multinomial with credible intervals in a Bayesian framework. This study provides a comprehensive review of election forensics. It examines the applicability and limitations of Benford's second-order test of conformity (using first two digits) and Hartigans' dip test of unimodality as baseline tests to statistically determine possible/suspected irregularities in Ghana's 2012 and 2020 electoral votes count.

The circumstance of a losing candidates failing to accept the outcome of election results has led to the loss of lives, properties, and relocation of people [10]. Election forensics has been used in many countries to test whether possible anomalies and irregularities exist in the election result using valid vote counts, e.g. [11] and [12]. Many countries have had their election results and processes tested, and good results and findings were produced in those research. Researchers have utilized a host of statistical methods to assess election results as indicators of election irregularities in several countries like Nigeria [13], Egypt [14], Afghanistan [15], Russia [16], [17], [18], Iran [19], [20]. Past statistical analyses have focused on different data reported by electoral commissions: voter turnout, votes earned by each candidate, and the number of invalid vote counts (rejected votes). Some authors have examined the combination of these detailed information on votes cast. The exploration can take one of these two approaches. The first approach assumes what ought to occur in an election free of irregularities and anomalies by the political parties involved; whereas the second adopts the reciprocal strategy and accepts what ought to happen if election results are tampered with. [21] assert that one statistical methodology used to examine data integrity relies on Benford's Law.

Election anomalies are irregularities or unpredictable events that occur before, during and after a voting process. Election irregularities can take many forms, including vote manipulation [22], [23], voting machine hacking [24] and voter suppression [25], [26], [27]. With the increased usage of computerized voting methods in recent years, concerns about the possibility of election irregularities have intensified. While these systems have various advantages, like enhanced speed and accuracy in voting, they also pose security risks such as hacking. Election anomalies are a serious problem in contemporary electoral systems because they have the ability to affect an election's outcome and erode public's trust in the electoral system. To create successful prevention and impact-mitigation techniques for election irregularities, further study is required to better understand their origins. A variety of methods has been developed to detect anomalies in election data, including but not limited to statistical analysis which entails employing statistical models to discover trends and discrepancies in election data that may suggest manipulation or interference [28], machine learning which includes employing algorithms to evaluate election data and discover irregularities [29], and blockchain technology which involves the use of decentralized and secure digital ledgers to record voting data and election results for rapid and efficient vote counting and results verification [30].

[11] relied on the Second-digit, 2BL mean developed by [17] to analyze the Bundestag elections in Unified Germany. The data on district-level results from German general elections spanning from 1990 to 2005 was used. Firstly, the vote count for each candidate was obtained at the district level. Secondly, the second-digit frequencies of all numerals were calculated. Lastly, a simple Pearson chi-square, $\chi^{2}$ test statistic was computed to identify a possible association between the observed and expected frequencies. In both 1990 and 2005, the standard frequencies significantly deviate from the observed frequencies. This implies a violation of Benford's Law, which indicates suspected anomalies and irregularities. A $\chi^{2}$ test statistic of 37.87 and 42.60 for 1990 and 2005, respectively, concluded that the distribution of the second digit does not conform to that of Benford, suggesting possible election anomalies. Though Germany's Western part recorded more violations than its Eastern counterparts, there was a revelation of minimal evidence of irregularities in connection to party votes from 1990 to 2005 in Unified Germany. Is there an association between foreign election observation, election anomalies, and post-election violence? Free and fair elections are the main aim of every democratic country's Electoral Commission. The presence of international observers from all walks of life plays a crucial role in maintaining peace and order after elections. [31] analyzed elections on the African continent using data from 1997 to 2009 in all African countries. The association between the response and independent variables was estimated by the Negative Binomial model other than a Poisson model due to the overdispersion exhibited by the dependent variable. The findings suggested that the probability of post-election violence increases with the presence of election anomalies and corrupts foreign observers. The results from matched samples and unmatched samples were not different, confirming the robustness of the test.

However, [32] combined both Benford's like Law (2BL) second-digit and the last digit mean (LastC) to detect election anomalies and irregularities in Russia with the use of vote counts digits. Since 2004 there have been widespread claims of election anomalies in Russian federal elections [12], [18] making Russia an ideal developed country to check for incidence of fraudulent polls to see statistical backings to these claims. With the help of district-level data from Russian federal elections, a randomization test was conducted to identify precincts known as UIKs in the Russian domain. The execution of the digits test (both the second and last digit) produced surprising results. For instance, both tests suggest that Putin's votes in 2004 and 2012 were not fraudulent, whilst Medvedev's votes in 2008 were adjudged to be fraudulent. [32] strongly argues that Putin's vote counts in 2012 were fraudulent as his analysis revealed that $\chi_{2BL}^{2}$ do not follow the distribution specified by Benford law. A tentative case study of most post-election conflicts in Africa is nothing worth writing about as it has been on record to be part of the continent's dark history. For example, the disputed 2007 general elections in Kenya ended in violence which took away 1,100 lives and had a whopping 350,000 citizens displaced [33]. [34] provided a comparative analysis of election forensic techniques such as the unimodality test, Zero Five Count Mean, skewness, kurtosis, Last Digit Mean, and Second Digit Mean to detect possible fraud in Georgia and Armenia parliamentary and presidential elections using precinct-level data. Apart from the dip test of unimodality, bootstrapping was used as a resampling procedure to generate 95% confidence intervals for the remaining tests. The conclusions from the election forensics adopted suggested several statistical anomalies and irregularities in the parliamentary and presidential elections between 2007 and 2016 in Georgia and Armenia.

While the Benford test can be beneficial for detecting anomalies in large datasets, it does have significant drawbacks. First, it may yield false positives or false negatives, especially in small datasets or datasets with non-uniform distributions [35], [36]. Second, the test implies that the data is independent and identically distributed, which may not always be the case in real-world applications [37]. Lastly, the test may be unable to identify more sophisticated kinds of fraud or manipulation involving electoral data [38]. Although the dip test is widely used, it has significant limitations. One limitation is that it assumes the dataset is unimodal, which may not always be the case in real-world applications [39]. Also, the dip test may be insensitive to tiny modes or modes that are close together [40]. Additionally, when employed with small or highly skewed datasets, the test may produce false positives or false negatives results [41], [42]. Even as the Hartigan dip test of unimodality and Benford second order test of conformity can be effective for identifying suspected fraud and anomalies in election numerical data, it should be used cautiously (as baseline tests) and in conjunction with other analytical techniques (finite mixture fraud models) to provide accurate and trustworthy results. Even though [38] argues that Benford Law has some limitations as an election forensic tool, when used and found to be significant, it raises some red flags about the electoral data integrity and hence can be used as a baseline test for further investigations to be conducted. Although Benford Law cannot be used as full proof of election anomaly or fraud, one major strength lies in its usage as a red flag that can prompt further investigation. Datasets may deviate from Benford's distribution for other reasons than manipulation and even then Benford Law can be used as a method of raising red flags [43]. Given these evidences from other parts of the world, it is then imperative to also check for suspected election irregularities and anomalies in the Ghanaian setting (with focus on the stronghold and swing regions since elections are won in Ghana primarily by winning in majority of the swing regions), using the Hartigan's dip and Benford tests (with special focus on the first two significant digits) as baseline tests; hence, the core of this research.

The remainder of the paper is organized as follows: Section 2 gives the review of existing methods of possible election anomaly detection. Section 3 discusses the data and the results of the specific application. Section 4 concludes the study and provide recommendations for further work.

## 2 Review of existing methods of election forensics

Some of the existing statistical techniques used in detecting possible or suspected election anomalies and irregularities that are key to this research are discussed in this section.

### 2.1 Benford second order test

Walter Mebane, a University of Michigan political scientist and statistician, was the first to use the second-digit Benford's law-test (2BL-test) in electoral forensics [44]. Although this technique is seen to be a straightforward method of detecting potential irregularities in election results, it is not thought to be perfect. In a 2011 research, political scientists Joseph Deckert, Mikhail Myagkov, and Peter C. Ordeshook asserted that when employed as a statistical indication of election fraud, Benford's law can produce deceptive outcomes [38]. [45] criticized their paper, criticizing their technique while acknowledging that utilizing Benford's formula to examine election data had significant limitations. In view of the above assertions on the applicability of Benford's Law, it is important to take note that for data analytic problems, a large deviation from Benford's Law suggests suspected irregularities and anomalies and should therefore be investigated further [46]. The second-order test is a good test to return compliant results for sets of data with omissions and errors [47], [48]. However, issues with the data that the second-order tests will find difficult to detect would not also be detectable using the usual descriptive summary statistics such as Skewness and Kurtosis.

For the Benford test, the hypothesis of interest is:

$H_{0}:Valid\;votes\;count\;follow\;the\;distribution\;specified\;by\;Benford$

$H_{1}:Valid\;votes\;count\;do\;not\;follow\;the\;distribution\;specified\;by\;Benford$

With a computed Benford statistic, rejecting the null hypothesis leads to the conclusion that there is a significant difference between observed and expected valid votes count, and hence elections were prone to possible anomalies.

The computation for the Lower and Upper bounds are respectively given by (1) and (2) as

(1) $$Lower\;Bound=PE-\left[Z_{\frac{\alpha }{2}}\times \sqrt{\frac{PE(1-PE)}{W}}\right]-\left(\frac{1}{2W}\right),$$

and

(2) $$Upper\;Bound=PE+\left[Z_{\frac{\alpha }{2}}\times \sqrt{\frac{PE(1-PE)}{W}}\right]+\left(\frac{1}{2W}\right),$$

where *PE*, *W* and *α* are quantile of the standard normal respectively. The presence of Benford's Law in certified election results data at hand is verified thoroughly by resorting to three (3) different tests.

I. **Benford Chi-Square test:** The goodness of fit test (Pearson Chi-Square) is well known to investigate whether a given set of data $Z_{1},Z_{2},\ldots ,Z_{n}$ fit a particular distribution function $Q_{0}$. Here, Benford's empirical distribution ${\overset{ˆ}{Q}}_{n}$ is compared to the samples $Q_{0}$. The assumption usually used is the asymptotic normality. The Benford second-order $\chi^{2}$ test statistic computed by (3) as
  (3) $$\chi_{Stat}^{2}=\sum_{k=10}^{99}\frac{{\left(f_{k}^{o}-f_{k}^{e}\right)}^{2}}{f_{k}^{e}},$$
  where $f_{k}^{o}$ is the count of the observed digit *k* and $f_{k}^{e}$ is the count of the expected digit *k*. For this underlying distribution where *k* possible digit combinations are considered, the critical value is given by $\chi_{Crit}^{2}=\chi_{k-1}^{2},\alpha$. For this study, the first two significant digits will be preferred because it captures more information; thus there are 90 possible digit combinations (10–99 inclusive) with a significance level of 0.05. Thus, the critical value for the test will be given by $\chi_{90-1,0.05}^{2}=\chi_{89,0.05}^{2}$. A comparison will then be made between a computed $\chi_{Stat}^{2}$ and the $\chi_{Crit}^{2}=112.022$. The null hypothesis of no significant difference between observed and expected valid vote count is rejected for large values of the Pearson $\chi_{Stat}^{2}$.
II. **Mean Absolute Deviation,***MAD***:** The *MAD* does not take into account the number of observations under study, *W* say. This makes it less sensitive to both small and large deviations as *W* is increased making it the best test to use for real-life data [49].
  Mathematically (4)gives the computation of the MAD,
  (4) $$MAD=\frac{\sum_{i=1}^{v}|P_{i}-PE_{i}|}{v},$$
  where, *v* is the number of bins that is equal to 90 for the first two digits, *P* is the observed proportion and *PE* is Benford's expected proportions.
III. **Mantissa Arc Test,***MAT***:** It calculates the digits of the numbers, and a comparison is made between the actual and the expected frequencies of Benford's law. *MAT* is the mathematical cornerstone of Benford's law and uses the mean vector of a set of mantissa distributed on a unit circle. For any given number *y*, the abscissa and ordinate are given respectively by (5) and (6) as
  (5) $$abscissa=\cos[2\pi \log_{10}(y_{i})mod1].$$
  (6) $$ordinate=\sin[2\pi \log_{10}(y_{i})mod1].$$
  When the mantissa set of numbers $y_{1},y_{2},\ldots ,y_{n}$ are distributed uniformly on a unit circle, the point (0,0) becomes the mean vector and we can make a conclusion that the data conforms to the distribution specified by Benford.
  The co-ordinates of the mean vector are given in (7) and (8) by
  (7) $$abscissa=\frac{\sum_{i=1}^{W}\cos[2\pi \log_{10}(y_{i})mod1]}{W},$$
  and
  (8) $$ordinate=\frac{\sum_{i=1}^{W}\sin[2\pi \log_{10}(y_{i})mod1]}{W},$$
  where *W* represents the number of records under consideration.
  The mean vector's length $L^{2}$ and the P-value are given respectively by
  (9) $$L^{2}={\left(abscissa\right)}^{2}+{\left(ordinate\right)}^{2}.$$
  and
  (10) $$P-value=1-\exp\left\{-L^{2}\times W\right\}.$$
  It can be inferred from (9) and (10) that as $L^{2}$ gets closer to 1 and *W* approaches infinity, the significant probability (P−value) approaches 1.

Table 1 summarizes the ranges and scores of Benford's law conformity test adopted from [48].

**Table 1:** Digits Range and conclusions for MAD values.

Digits	Range	Conformity conclusion
First Digit	0.000 to 0.006	Close
	0.006 to 0.012	Acceptable
	0.012 to 0.015	Marginally Acceptable
	Above 0.015	Nonconformity

Second Digit	0.000 to 0.008	Close
	0.008 to 0.010	Acceptable
	0.010 to 0.012	Marginally Acceptable
	Above 0.012	Nonconformity

First-Two Digit	0.000 to 0.012	Close
	0.012 to 0.018	Acceptable
	0.018 to 0.022	Marginally Acceptable
	Above 0.022	Nonconformity

### 2.2 Data diagnostics using Benford's law

[50] assert that “If W∼U(a,b) where *a* and *b* are real numbers satisfying a<b. If the interval $\left(10^{a},10^{b}\right)$ covers an integer number of orders of magnitude, then the first significant digit of the random variable $T=10^{W}$ satisfies Benford's Law exactly”. The lemma can be interpreted simply as the specific probability distribution of all the digits under consideration of the possible values of *T* that constitutes a Benford's set. It is to be noted here that *T* is a stochastic variable and just one number cannot comprise a Benford.

For any given set of numbers, Benford's Law is said to be satisfied if the first significant digit says, $G_{1}$ of the number follows the following given probability distribution specified in (11) by;

(11) $$Pr(G_{1}=g_{1})=\log_{10}\left(1+\frac{1}{g_{1}}\right),\;\;\;\;g_{1}\in \{1,\ldots ,9\},$$

where *Pr* designates the probability of observing the event $\left(G_{1}=g_{1}\right)$.

Traditionally, Benford's Law can be viewed as

$$Pr(G_{1}=g_{1})=\log_{10}(g_{1}+1)-\log_{10}(g_{1})=\log_{10}\left(\frac{g_{1}+1}{g_{1}}\right)=\log_{10}\left(1+\frac{1}{g_{1}}\right).$$

In general, the distribution of the first *m* significant digits, $g_{1},g_{2},\ldots ,g_{m}$ is specified by (12) as,

(12) $$Pr(G_{1}=g_{1},G_{2}=g_{2},\ldots ,G_{m}=g_{k})=\log\left[1+{\left(\sum_{j=1}^{m}g_{j}\times 10^{m-j}\right)}^{-1}\right],$$

for $g_{1}=1,2,3,\ldots ,9$ and $g_{2},\ldots ,g_{m}=0,1,2,3,\ldots ,9$

### 2.3 Benford's law mechanism

Assume we consider the random variable $Z=10^{Y}$ where *Y* is a Uniform distribution on the interval (0,1). That is to say Y∼U(0,1) with expectation $\frac{1}{2}$ and variance $\frac{1}{12}$. Suppose we choose a value for *Z* which has a significant digit $g_{1}\in \{1,\ldots ,9\}$, then the random variable *Z* will automatically be in the interval in (13).

(13) $$10^{k}g_{1}\leq Z\leq 10^{k}(g_{1}+1),$$

for some integer *k*.

Taking logarithm to the base 10 of (13) yields (14) as

(14) $$k+\log_{10}g_{1}\leq \log_{10}Z<k+\log_{10}(g_{1}+1).$$

The length of the interval in (14) is given by (15) as

(15) $$\log_{10}(g_{1}+1)-\log_{10}g_{1}=\log_{10}\left(\frac{g_{1}+1}{g_{1}}\right)=\log_{10}\left(1+\frac{1}{g_{1}}\right),$$

which is just the probability that *Z* has first digit $g_{1}$.

This logic is an indication that if a stochastic variable Y∼U(0,1) then, $Z=10^{Y}$ satisfies Benford's law. Therefore, a sure way to construct numbers that will closely conform to Benford's law is to generate numbers from a uniformly distributed random variable on the interval (0,1) with the help of a random number generator and exponentiate the random numbers generated with $10^{Y}$. In practice, perfect conformity to Benford's law for real data may not be possible. However, conformity to Benford's Law does not signal that the data is omission-free but nonconformity does signal an issue with data integrity.

### 2.4 Dip test of unimodality

[39] asserts that “For any given empirical cumulative distribution function and the set of the uni-modal distributions *μ*, the *cdf* of the set *μ* are well characterized: they are convex on an interval $\left[-\infty ,x_{l}\right]$, then constant on $\left[x_{l},x_{u}\right]$ and concave on $\left[x_{u},+\infty \right]$”.

The distribution of the voters turnout only need not be uni-modal to give strong evidence of anomaly free elections, but also the distribution of the winners' share in an election should be uni-modal likewise [51].

For the dip test of unimodality, we test the hypotheses:

$$H_{0}:The\;distribution\;of\;valid\;votes\;cast\;is\;unimodal$$

$$H_{1}:The\;distribution\;of\;valid\;votes\;cast\;is\;not\;unimodal$$

The adoption of Hartigans' dip test for unimodality arises from the argument that if the empirical distribution of the proportion of votes cast is not uni-modal (thus, if it has multiple peaks), then there is a possible indication of election anomalies or irregularities. The dip test developed by [40] gives a measure of the distance between the set of uni-modal distributions and empirical cumulative distributions.

Following [40], we let *F* be any arbitrary probability distribution function of interest. Then if we let D(F)=e only if there exists a non-decreasing function *H* such that for some $x_{l}\leq x_{u}$,

(i) *H* is the Greatest Convex Minorant (GCM) of F+e in $\left(-\infty ,x_{l}\right)$.
(ii) *H* has a constant maximum slope in $\left(x_{l},x_{u}\right)$.
(iii) *H* is the Least Concave Majorant (LCM) of F−e in $\left[x_{u},\infty \right)$.
(iv) $e=sup_{x\notin (x_{l},x_{u})}|F(x)-H(x)|\geq sup_{x\in (x_{l},x_{u})}|F(x)-H(x)|$.

Here, D(F) is the value of *e* such that any further decrease forces the string out of its unimodal shape. We can deduce that the dip automatically determines $\left[x_{l},x_{u}\right]$, the modal interval where $x_{l}$ is the lower modal limit, and $x_{u}$ is the upper modal limit. Since the dip test is much superior to the likelihood ratio test in detecting election anomalies and irregularities, we shall therefore stick to the employment of Hartigans' dip test in this study other than the likelihood ratio test. Large significant probability values give justification to retain the null hypothesis of unimodality. Hence, in the absence of suspected election anomalies and irregularities, we thus expect the p-value value of the dip to be greater than 0.05.

### 2.5 Second-digit mean, 2BL

The second digit in each count to which a particular test is applied is referred to as 2BL. In the presence of possible problematic elections, the distribution that the second digits exhibits should deviate from the distribution implied by Benford's Law [52]. Hence, in the absence of election anomalies and irregularities, we thus expect 2BL of value to be equal to 4.187, that is 2BL=4.187.

### 2.6 Bi-modality coefficient

The Bi-modality Coefficient (BC) given by (16) is one of the numerous empirical methods in literature with the assumption of a distribution exhibiting bi-modality to have low kurtosis, high skewness, or even both [42]. The *BC* values which are a function of sample size, skewness given by (17) and kurtosis given by (18) are very easy to compute.

The value of the *BC* is computed as

(16) $$BC=\frac{k_{3}^{2}+1}{k_{4}+3\times \left[\frac{{\left(q-1\right)}^{2}}{\left(q-2)(q-3\right)}\right]},$$

where *q* is the size of the sample, $k_{3}$ is the skewness and $k_{4}$ is the excess kurtosis for the available data. Due to the sensitivity of skewness and kurtosis to sample bias, we have to likewise correct for sample bias using

(17) $$k_{3}=\frac{\sqrt{q(q-1)}}{\left(q-2\right)}\left\{\frac{\left(\frac{1}{q}\right)\sum_{j=1}^{q}{\left(y_{i}-\overset{¯}{y}\right)}^{3}}{{\left(\sqrt{\left(\frac{1}{q}\right)\sum_{j=1}^{q}{\left(y_{i}-\overset{¯}{y}\right)}^{2}}\right)}^{3}}\right\}.$$

and

(18) $$k_{4}=\frac{\left(q-1\right)}{\left(q-2)(q-3\right)}\cdot \left[(q+1)\left\{\frac{\left(\frac{1}{q}\right)\sum_{j=1}^{q}{\left(y_{i}-\overset{¯}{y}\right)}^{4}}{{\left(\left(\frac{1}{q}\right)\sum_{j=1}^{q}{\left(y_{i}-\overset{¯}{y}\right)}^{2}\right)}^{2}}\right\}-3(q-1)\right].$$

If BC≤0.555, the distribution of the given data is considered unimodal if not a bimodal or multimodal distribution is assumed. A higher level of significance leads to a higher probability of identifying data exhibiting unimodality compared to those of multimodality and vice versa. [42] also postulate that even though the Hartigans' dip statistic (HDS) is more useful than the *BC*, the *HDS* is very subjective and difficult to use in the sense that researchers have to select an appropriate level of significance based on the size of the sample under consideration. It is therefore prudent for researchers to choose an appropriate significance level to avoid both Type I and Type II errors.

### 2.7 Skewness

If arguments are raised in favour of unimodality then we expect that the distribution of voters' turnout proportion should be approximately normal and the Skewness should be approximately zero [53]. There may be problems with election results if Skewness differs significantly from zero. Most widely used Skewness index, Skew is given by (19) as

(19) $$Skew=\frac{m_{3}}{m_{2}^{\frac{3}{2}}},$$

where $m_{3}=\frac{\sum_{i=1}^{n}{\left(y_{i}-\bar{y}\right)}^{3}}{n}$ and $m_{2}=\frac{\sum_{i=1}^{n}{\left(y_{i}-\bar{y}\right)}^{2}}{n}$. Here, $m_{3}$ is the third moment and $m_{2}$ is the variance. In the absence of suspected election anomalies and irregularities, we expect the Skewness value to be approximately equal to 0, that is Skew=0.

### 2.8 Kurtosis

If arguments are raised in favour of unimodality then we expect that the distribution of voters turnout proportion should be normal and the kurtosis should be approximately three (3). There may be problems with election results if kurtosis differs significantly from the value of three. In the absence of possible election anomalies, we expect the kurtosis value to be approximately 3, that is Kurt≈3. This implies that the kurtosis of a rigged election either substantially exceeds 3 or substantially falls below 3. The coefficient of Kurtosis is given by (20) as:

(20) $$Kurt=\frac{m_{4}}{m_{2}^{2}},$$

where $m_{4}=\frac{\sum_{i=1}^{n}{\left(y_{i}-\bar{y}\right)}^{4}}{n}$ is the fourth moment and $m_{2}$ is defined as above in skewness.

### 2.9 Last-digit mean

The last digit in each count to which a particular test is applied is referred to as LastC. As a scenario, considering a vote of count “5678” per say, we observe that 8 is the last digit. In a problematic free election we expect a uniform distribution for the last digits. That is the say that the probability of each of the ten digits (0,1,2,3,4,5,6,7,8,9) occurring is $\frac{1}{10}=0.1$. In instances where the last digits occur with such probabilities, the average of the last digits is given by equation (21) as

(21) $${\bar{X}}_{k}=\frac{1}{10}\sum_{k=0}^{k=9}k=\frac{45}{10}=4.5$$

Hence, in the absence of possible election anomalies and irregularities, we thus expect the value of the Last digit mean to be equal to 4.5, that is LastC=4.5.

### 2.10 Summary of tests for election anomaly detection

Table 2 summarizes various statistical methods in the literature used in election anomaly detection.

**Table 2:** Distribution and Digit tests of Election Anomaly Detection.

Test	Value in the absence of anomaly
Dip Test, *DipT*	*P* − *value* > 0.05
Benford Test, $\chi_{stat}^{2}$	≤112.022
Second-digit mean, 2*BL*	4.187
Last-digit mean , *LastC*	4.5
Skewness, *Skew*	≈0
Kurtosis, *Kurt*	≈3
Bimodality Coefficient, *BC*	≤0.555

Source: A Guide to Election Forensics, 2015 [53]

For the purpose of this study equations (22) and (23) will be used as a guide in assessing anomaly percent rates,

(22) $$Non-Anomalous\;Detection\;Rate,\;(NADR)=\frac{Number\;of\;Anomalous\;free\;Subsets}{Total\;Number\;of\;Subsets}\times 100\text{\%}.$$

The Anomalous Detection Rate, (ADR) is computed accordingly as;

(23) $$Anomalous\;Detection\;Rate,\;(ADR)=\frac{Number\;of\;Anomalous\;Subsets}{Total\;Number\;of\;Subsets}\times 100\text{\%}.$$

## 3 Results and discussion

The study made use of secondary data comprising of *2012* and *2020* Presidential election certified results in Ghana based on the *275* constituencies. The data used for the analysis of the study was obtained from the Electoral Commission, EC of Ghana. The data obtained were grouped into three *(3)* categories; that is, the election results of the NPP, NDC, and Other political parties (i.e. all the other political parties with the exemption of NPP and NDC). The two regions selected in our criteria as stronghold are Ashanti and Volta. Since there have been alleged claims of over-voting and cheating in the stronghold (Ashanti and Volta) of NPP and NDC, respectively, our primary focus was on these two regions. Elections in Ghana are also won primarily by winning in all or most swing regions. Thus, checking for possible anomalies and irregularities in these regions is justifiable. A comparative analysis of election forensics was made between the Benford second-order conformity test (with particular emphasis on the first two digits) and the Hartigans' dip test of unimodality to detect the existence of possible or suspected election anomalies and irregularities. The codes for the study are available on GitHub. The GitHub repository can be found at https://github.com/Agyemang1z/Election-Forensics. For brevity and ease of presentation, the dip plots of the two stronghold regions (Ashanti and Volta) and the three swing regions (Greater Accra, Central, and Western) of NPP and NDC in the 2020 presidential elections are displayed in Fig. 1.

**Figure 1:** 2020 dip plots of stronghold and swing regions in Ghana.

From Fig. 1, unimodality is observed by a single peak, whilst double and multiple peaks exhibit bi-modality and multimodality. It is worth knowing that the plots of unimodality though an informal test of anomaly detection, are unreliable because it is likely to be influenced by bandwidth, as a poorly chosen bandwidth can lead to an undesirable transformation of the density plot. The formal test, Hartigan's dip test of unimodality, is used in the analysis of possible election anomaly or manipulation.

### 3.1 Assessing Benford's minimal assumptions in stronghold and swing regions

The minimal conditions required for the application of Benford's law for first digit analysis include large data sets whose numbers combine multiple distributions, cover several orders of magnitude, and where the mean is greater than the median with a positive skew [38], [54], [55], [56], [57]. However, if these conditions are violated, second-digit analysis should be resorted to instead [44], [45], [58]. At both stronghold and swing regional levels, *417* aggregated data points from *15,835* polling stations in *2012* and *17,881* polling stations in *2020* were used for the study. *139* aggregated data points (representing the vote counts in each of the constituencies in both stronghold and swing regions) for each party (47 for Ashanti region, 18 for Volta region, 34 for Greater Accra region, 23 for Central region and 17 for Western region) which makes it a large data set enough (sufficiently large sample size per central limit theorem). It was also observed that the valid vote counts of both NPP and NDC in stronghold and swing regions cover several orders of magnitude (for brevity, one of the stronghold regions illustrated in Fig. 3 and Fig. 4. Furthermore, since the Other political parties make less than 3% of the votes count in Ghana, their departure from Benford distribution will not give something worthwhile but it was included in the analysis as a baseline guide. From Table 3, it can be observed that not all the mean number of votes are greater than their corresponding median number of votes at the various regional levels. It can thus be concluded that Ghana's electoral data for the analysis of this study is sufficiently large enough, cover several orders of magnitude but not all the mean number of votes count in respective stronghold and swing regions are greater than the median number of votes count with a positive skew as evident in Table 3. With the above justification, this study resorted to the Benford's first-two significant digits analysis as a baseline test in checking for election fraud, anomalies and irregularities since it captures more information - 90 possible digit combinations (10–99 inclusive) compared to the second digits - 10 possible digit combinations (0-9 inclusive) as proposed by [44], [45], [58].

**Table 3:** Summary of Coefficient of Skewness output in Stronghold and Swing Regions.

Regional votes count	Parties	2012 elections			2020 elections		
		Mean	Median	Skewness	Mean	Median	Skewness
Ashanti	NPP	32577.7	31710	0.2961	38209.09	35144	0.6246
	NDC	13034.38	11239	2.2326	13896.96	12534	2.3191

Volta	NPP	4274.96	2851	1.0452	5577.72	4106.5	1.4465
	NDC	28255.42	22456	1.7944	33704.89	32648.5	1.4010

Greater Accra	NPP	29699.62	30862	-0.0531	36769.97	37795	0.1508
	NDC	33110.32	31849	0.6909	39014.38	36245.5	0.7609

Central	NPP	18701.52	18834	0.1839	26687.13	26629	1.4117
	NDC	21407.57	21999	0.1773	23426.48	21209	1.2437

Western	NPP	18019.88	17475	0.4825	25871.41	25095	0.8367
	NDC	22392.04	19857	0.3128	23444.06	19942	1.0464

### 3.2 Assessing homogeneity assumption in stronghold and swing regions

Even though bimodal or multimodal distribution, however, does not necessarily indicate manipulation, it does pose some threat to the authenticity of the data. [59] highlighted that bimodal distributions can also result from combining observations with covariates correlating with the turnout (e.g., income or education). To rule out alternative reasons beyond election anomalies, the authors recommended accounting for unit homogeneity and, if possible, comparing the distributions over time to detect non-uniform changes in the turnout levels. The homogeneity assumption was accounted for in this study by the use of the permutation test, a non-parametric test that is used to determine whether two or more groups of data come from the same population. This test involves randomly permuting the data among the respective groups and calculating the p-value as the proportion of simulated statistics that are more extreme than the observed statistic. With *10,000* permutations for each stronghold regional test and all p-values (>0.05) as evident in Table 4, we retain the null hypothesis of homogeneity (under the assumption of no difference between the three groups- NPP, NDC and other political parties) and conclude that the null distribution is symmetric and centred around zero. In effect, the homogeneity assumption is valid and the dip test is appropriate for the analysis of Ghana's 2012 and 2020 electoral dataset.

**Table 4:** Summary of P-values of Permutation Test in Stronghold and Swing Regions.

Year	Parties	Stronghold regions		Swing regions		
		Ashanti	Volta	Greater Accra	Central	Western
2012 Elections	(NPP, NDC,Others)	0.965	0.052	0.999	0.993	0.977
2020 Elections	(NPP, NDC,Others)	0.924	0.112	0.998	0.999	0.987

### 3.3 A case study of the 2016 presidential elections

Even though the 2016 presidential elections held in Ghana were not challenged in court, it is essential to conduct a thorough analysis to ensure the integrity and fairness of the electoral process.

From Table 5, the Hartigans' dip test of unimodality suggests that the distribution of voters proportion for NPP, NDC, and Other political parties in both stronghold and swing regions are unimodal (p-values >0.05) indicating possible absence of anomalies and irregularities. Thus, no possible red flags are raised by the dip test. The Benford test however concluded that the distribution of valid voters for $NDC_{Ashanti}$, $NPP_{Volta}$ and $NPP_{GreaterAccra}$ are not unimodal (with p-values <0.05) confirming the suspected presence of anomalies and irregularities worth investigating. The significant deviations for the NDC in the Ashanti region and the NPP in the Volta region may not due to any manipulation but may be due to the fact that very few votes were obtained by respective parties in their opposition's stronghold. However, the significant deviation of NPP in the Greater Accra region therefore raise red flags for further investigation.

**Table 5:** Hartigan Dip Test and Benford Test of conformity (2016 Elections).

Swing regions	Parties	Dip test		Benford test	
		Dip Statistic	P-value	*χ*^2^ Test Statistic	P-value
Ashanti	NPP	0.0456	0.6670	94.204	0.3327
	NDC	0.0549	0.3395	145.690	0.0001

Volta	NPP	0.0622	0.6100	140.390	0.0004
	NDC	0.0506	0.9095	83.350	0.6489

Greater Accra	NPP	0.0646	0.3170	146.400	0.0001
	NDC	0.0601	0.4335	108.470	0.0787

Central	NPP	0.0844	0.1785	94.548	0.3237
	NDC	0.0558	0.8545	88.853	0.4844

Western	NPP	0.0554	0.7950	60.866	0.9902
	NDC	0.0712	0.3420	79.103	0.7645

### 3.4 Calculating ashanti region dip test statistic for NPP, NDC and others

With n=47 constituencies under consideration in Ashanti region, we observe from Fig. 2(a) that the modal interval for NPP is $\left(x_{l},x_{u})=[x_{22},x_{30}=(30992,35417)\right]$ and the *GCM* and *LCM* have 3 and 4 nodes (shown in red and blue circles respectively) inside $\left(x_{l},x_{u}\right)$. Likewise, we observe from Fig. 2(b) that the modal interval for NDC is $\left(x_{l},x_{u})=[x_{16},x_{31}=(10144,12998)\right]$ and the *GCM* and *LCM* have 4 and 3 nodes (shown in red and blue circles respectively) inside $\left(x_{l},x_{u}\right)$.

**Figure 2:** Plot of 2012 Empirical cdf in Ashanti Region for NPP and NDC.

Now, beginning with an R Studio generated dip loop, $D_{loop}$ of *3.920833*, the dip test statistic for NPP in Ashanti region is given by:

$$Dip_{NPP}=\frac{D_{loop}}{2n}=\frac{3.920833}{2\times 47}=0.0417$$

Likewise, with a $D_{loop}$ of *5.105108*, the dip statistic of NDC in Ashanti is given by:

$$Dip_{NDC}=\frac{D_{loop}}{2n}=\frac{5.10508}{2\times 47}=0.0543$$

Finally, with a $D_{loop}$ of *3.615385*, the dip statistic of Other Political Parties in Ashanti region is given by:

$$Dip_{Others}=\frac{D_{loop}}{2n}=\frac{3.615385}{2\times 47}=0.0385$$

We use similar arguments to arrive at the dip statistic for all the other regions considered in the study.

From Table 6, for the stronghold regions under consideration, the Hartigans' dip test of unimodality suggests that the distribution of voters proportion for NPP, NDC, and Other political parties in both Ashanti and Volta regions are unimodal (p-values >0.05) indicating the possible absence of anomalies and irregularities.

**Table 6:** Summary of unimodality Test output (Stronghold Regions).

Region	Party	2012 elections		Modal interval [*x*_*l*_,*x*_*u*_]
		Dip Test Statistic	P-value	
Ashanti	NPP	0.0417	0.8175	[30992,35417]
	NDC	0.0543	0.3510	[10144,12998]
	Others	0.0385	0.9090	[366,380]

Volta	NPP	0.0751	0.2625	[802,2683]
	NDC	0.0672	0.4565	[20819,22571]
	Others	0.0597	0.6650	[397,408]

Also from Table 7, for the three swing regions, the Hartigans' dip test of unimodality concluded that the distribution of valid voters proportions for NPP, NDC, and Other Political parties in the Greater Accra, Central, and Western regions are unimodal (with p-values >0.05) confirming the possible absence of anomalies and irregularities. This indicates that elections were possibly conducted in an anomalous free manner.

**Table 7:** Summary of unimodality Test output (Swing Regions).

Region	Party	2012 elections		Modal interval [*x*_*l*_,*x*_*u*_]
		Dip Test Statistic	P-value	
Greater Accra	NPP	0.0422	0.9500	[33424,35242]
	NDC	0.0421	0.9460	[34802,36451]
	Others	0.0574	0.5160	[508,566]

Central	NPP	0.0735	0.7255	[9947,15339]
	NDC	0.0532	0.8970	[21228,23509]
	Others	0.0455	0.9815	[584,616]

Western	NPP	0.0502	0.9070	[11473,12030]
	NDC	0.0566	0.7425	[18928,19947]
	Others	0.0441	0.9795	[573,578]

The Non-Anomalous Detection Rate of the Hartigans' dip test of unimodality for 2012, ($NADR_{2012Dip}$) is computed as

$$NADR_{2012Dip}=\frac{15}{15}\times 100\text{\%}=100\text{\%}$$

This suggests that per the findings of Hartigans' dip test of unimodality, there were 0% suspected anomalies or irregularities in both the stronghold and swing regions.

For brevity and ease of presentation, we display the Benford plots of NPP 2012 Election results in the Ashanti region and NDC 2012 Election results in the Volta region.

From Fig. 3 and Fig. 4, the second-order digits distribution plots are of principal interest. The first two digits are shown on the *abscissa-axis* and their frequency of occurrence is depicted on the *ordinate-axis*. It is usually based on sorting the data and plotting the differences. Benford's second-order test was then applied to the 2012 certified election results data from the Election Commission of Ghana, and non-conformance always signals an abnormal issue related to the integrity of the data. The fit of the observed proportions to that of expected (Benford's) proportion is visually fascinating, as depicted by both figures. We observe from the probability distributions of various stronghold regions that for a host of the higher (60 and above) - first-two significant digits combinations, the deviation between the observed and Benford's proportions is just a minute percentage.

**Figure 3:** Plot of NPP 2012 Benford second order test in Ashanti Region.

**Figure 4:** Plot of NDC 2012 Benford second order test in Volta Region.

For the stronghold regions, a computed $\chi^{2}$ test statistic value of *120.720* and *131.540* (from Table 8 highlighted in red) for NDC and Other political parties respectively in Ashanti region exceeded the $\chi_{crit}^{2}=112.022$ indicating non-conformity to Benford's Law. This, in turn, suggests that elections were conducted in a possible anomalous manner to either go for (an anomaly in favour of NPP) or against (anomaly against NDC) since the Ashanti region is the stronghold of NPP. Benford's test of conformity further revealed that except for NDC and other Political parties in the Ashanti region, elections were possibly conducted fairly in the two stronghold regions for all political fronts involved in the 2012 presidential elections (with computed $\chi^{2}$ test statistic values of *80.829*, *79.461*, *72.466* and *111.700* from Table 8 for $Ash_{NPP}$, $Volta_{NPP}$, $Volta_{NDC}$ and $Volta_{Others}$ respectively) with Volta region being likely anomalous free stronghold region in the 2012 Presidential elections held.

**Table 8:** Benford's Test output (Stronghold Regions).

Region	Party	2012 elections		MAD	P-value
		*χ*^2^ Test Statistic	MATS		
Ashanti	NPP	80.8290	0.1506	0.0115	0.7197
	NDC	120.7202	0.2093	0.0143	0.01422
	Others	131.5404	0.4360	0.0138	0.0023

Volta	NPP	79.4611	0.0135	0.0142	0.7555
	NDC	72.4663	0.1888	0.0143	0.8988
	Others	111.7002	0.0853	0.0160	0.05214

For the swing regions, Benford's test of conformity revealed that except for election results of other political parties in Greater Accra, Central and Western (with computed $\chi^{2}$ test statistic values of *176.1405*, *118.1002* and *139.2505* from Table 9 for $Accra_{Others}$, $Central_{Others}$ and $Western_{Others}$ respectively) where their computed Pearson test statistic exceeded the critical threshold value of *112.022*, elections were possibly conducted fairly in all the three swing regions for all political parties involved in the December 2012 electoral process in Ghana.

**Table 9:** Benford's Test output (Swing Regions).

Region	Party	2012 elections		MAD	P-value
		*χ*^2^ Test Statistic	MATS		
Greater Accra	NPP	106.5101	0.3520	0.0157	0.0995
	NDC	89.7863	0.4736	0.0148	0.4567
	Others	176.1405	0.6272	0.0172	0.0010

Central	NPP	82.9728	0.0779	0.0141	0.6599
	NDC	62.0296	0.4989	0.0139	0.9868
	Others	118.1002	0.4174	0.0169	0.0212

Western	NPP	55.6379	0.1719	0.0135	0.9978
	NDC	89.3763	0.2867	0.0143	0.4689
	Others	139.2505	0.2484	0.0160	0.0005

The Non-Anomalous Detection Rate of the Benford Second-Order test of conformity for 2012 ($NADR_{2012Benford}$) is computed as

$$NADR_{2012Benford}=\frac{10}{15}\times 100\text{\%}=66.67\text{\%}$$

This suggests that per the findings of the Benford Second-Order test of conformity, there was a 33.33% suspected anomaly or irregularities in both the stronghold and swing regions in the 2012 Presidential election held in Ghana.

The Overall Non-Anomalous Detection Rate of the two tests ($NADR_{2012Overall}$) for the 2012 Presidential elections is computed as

$$NADR_{2012Overall}=\frac{25}{30}\times 100\text{\%}=83.33\text{\%}$$

This suggests that from the analyses of both the Hartigans' dip test of unimodality and Benford Second-Order test of Conformity, there was a 16.67% suspected anomalies or irregularities in both the stronghold and swing regions in the 2012 Presidential election conducted in Ghana.

For the stronghold regions, the Hartigans' dip test of unimodality suggests that the distribution of voters proportion for NPP, NDC, and Other political parties in both Ashanti and Volta regions are unimodal (p-values >0.05), indicating a possibility of absence of anomalies and irregularities in the 2020 Presidential elections in Ghana as evident in Table 10.

**Table 10:** Summary of unimodality Test output (Stronghold Regions).

Region	Party	2020 elections		Modal interval [*x*_*l*_,*x*_*u*_]
		Dip Test Statistic	P-value	
Ashanti	NPP	0.0424	0.7795	[19224,29125]
	NDC	0.0319	0.9920	[12290,14721]
	Others	0.0428	0.7950	[213,252]

Volta	NPP	0.0962	0.1550	[3687,4186]
	NDC	0.0829	0.3740	[32229,33542]
	Others	0.0507	0.9885	[461, 473]

For the swing regions, the Hartigans' dip test of unimodality concluded that the distribution of valid voters proportion of NPP, NDC, and Other Political Parties in the Greater Accra, Central, and Western regions are unimodal (p-values > 0.05), suggesting a possible absence of anomalies and irregularities as seen in Table 11. This is an indication that elections were possibly conducted in an anomalous free manner and the data integrity was not perhaps tempered with.

**Table 11:** Summary of unimodality Test output (Swing Regions).

Region	Party	2020 elections		Modal interval [*x*_*l*_,*x*_*u*_]
		Dip Test Statistic	P-value	
Greater Accra	NPP	0.0322	0.9983	[37473,41485]
	NDC	0.0538	0.6210	[34555,38270]
	Others	0.0428	0.9390	[558,882]

Central	NPP	0.0523	0.9150	[26629,27670]
	NDC	0.9050	0.0529	[19163,21338]
	Others	0.0869	0.1695	[536,751]

Western	NPP	0.0602	0.8880	[23847,26396]
	NDC	0.3470	0.0859	[9254,11798]
	Others	0.0563	0.9650	[1359,1481]

The Non-Anomalous Detection Rate of the Hartigans' dip test of unimodality for 2020 elections data is the same as for the 2012 elections, as discussed above. Hence, there was a 0% suspected or possible anomaly or irregularities in both the stronghold and swing regions.

From Table 12, small values of Pearson's $\chi^{2}$ test statistic for all Political Parties in the two stronghold regions compared to the indicated critical value of *112.022* led to the conclusion of compliance to the distribution specified by Benford's Law. Thus, valid vote counts for all Political Parties in the 2020 Presidential elections in both the Ashanti and Volta regions are therefore not prone to possible manipulation, anomalies and irregularities.

**Table 12:** Benford Test output (Stronghold Regions).

Region	Party	2020 elections		MAD	P-value
		*χ*^2^ Test Statistic	MATS		
Ashanti	NPP	79.9510	0.1324	0.0118	0.7429
	NDC	93.0970	0.2625	0.0126	0.3623
	Others	109.5400	0.2379	0.0128	0.0689

Volta	NPP	93.1530	0.1645	0.0175	0.3608
	NDC	99.2930	0.1244	0.0168	0.2138
	Others	98.1460	0.1578	0.0171	0.2380

Likewise from Table 13, the Benford's Second Order test of Conformity further revealed that elections were possibly conducted in an anomalous free manner (with Pearson $\chi_{Stat}^{2}<112.022$) in all the three swing regions for all Political Parties involved in the December 2020 electoral process. This indicates that the observed frequencies of valid votes cast did not differ significantly from the expected frequencies specified by Benford's Law.

**Table 13:** Benford's Test output (Swing Regions).

Region	Party	2020 elections		MAD	P-value
		*χ*^2^ Test Statistic	MATS		
Greater Accra	NPP	93.9220	0.2338	0.0139	0.3401
	NDC	107.1700	0.4260	0.0157	0.4009
	Others	94.2570	0.2370	0.0153	0.3313

Central	NPP	62.6350	0.4691	0.0151	0.9847
	NDC	61.6300	0.3748	0.0147	0.9880
	Others	83.7470	0.1981	0.0160	0.6374

Western	NPP	56.6050	0.4466	0.0158	0.9971
	NDC	83.8230	0.0797	0.0173	0.6352
	Others	77.7290	0.0169	0.0168	0.7975

The Non-Anomalous Detection Rate of the Benford Second-Order test of Conformity for 2020 ($NADR_{2020Benford}$) is computed as

$$NADR_{2020Benford}=\frac{15}{15}\times 100\text{\%}=100\text{\%}$$

This suggests that per the analysis of the Benford Second-Order test of Conformity, there was a 0% suspected anomalies or irregularities in both the stronghold and swing regions in the 2020 Presidential election held in Ghana.

The Overall Non-Anomalous Detection Rate of the two tests for the 2020 ($NADR_{2020Overall}$) Presidential elections is computed as

$$NADR_{2020Overall}=\frac{30}{30}\times 100\text{\%}=100\text{\%}$$

This suggests that from the analyses of both the Hartigans' dip test of unimodality and Benford Second-Order test of Conformity, there was a 0% suspected anomalies or irregularities in both the stronghold and swing regions in the 2020 Presidential elections conducted in Ghana.

## 4 Conclusions and recommendations

Election anomaly detection is an important part of guaranteeing fair and free elections. Researchers have been investigating several strategies for detecting anomalies in election data, with the goal of assuring election results' accuracy, reliability, and transparency. Even though researchers like [38] argue that Benford Law when used as an election forensic in detecting anomaly or fraud is problematic, when used and found to be significant, it raises some red flags about the electoral data integrity and hence can be used as a baseline test for further investigations to be conducted. In this study, we resorted to exploring election forensic techniques such as the Hartigans' dip test of unimodality and Benford second order (with the application of the first two digits) test of conformity to statistically detect the existence of suspected or possible anomalies of valid votes count in the 2012 and 2020 Presidential elections held in Ghana. A comparative analysis of these two methods was then carried out. The contradictory conclusions from the two election forensics considered for the study of the 2012 valid votes count give a suspicion of possible irregularities and anomalies in the presidential election results (stronghold and swing regions) in Ghana (with an overall 16.67% suspected anomalies), which is subject to further investigation. This indicates some curiosities in the 2012 presidential election data worth unveiling. However, for the election forensics analysis of 2020 valid votes count, there was a perfect agreement between both tests, concluding a 0% suspected or possible anomalous elections. This indicates that the observed frequencies of valid votes count did not differ significantly from the expected frequencies specified by Benford's Law. This led to the conclusion of compliance with the distribution specified by Benford's Law. Thus, valid vote counts for all political parties in the 2020 Presidential elections in both the stronghold and swing regions are, therefore, not prone to suspected manipulation, anomalies and irregularities. The results of the 2020 anomaly detection for both Benford's Second-order test (using the first two digits) and Hartigans' dip test of unimodality are in perfect conformity with another study by [9] who made use of a Dirichlet Bayesian approach with credible intervals to reach similar conclusion. Likewise, the results of the 2020 presidential election anomaly detection also conform to the research by [8] who resorted to the applicability of digital frequency based analysis in election anomaly detection. The findings of this study suggest that the electoral process produced possible anomalous data in the 2012 presidential election results, whilst possible non-anomalous data was produced in the 2020 presidential election results of valid votes count. The study, therefore, recommended that for deeper statistical data analysis on election anomaly detection, researchers should start with Benford's second-order test of conformity and Hartigans' dip test of unimodality as baseline tests and progressively dig deeper into the application of finite mixture fraud models and machine learning techniques. More research is needed to increase the accuracy and reliability of these election forensic techniques as well as to ensure that election results are transparent and trustworthy. To conclude, election anomaly detection research plays an important role in ensuring fairness and integrity of democratic processes. To identify anomalies in election data, a variety of statistical and computational techniques have been developed, including Benford's Law, the dip test, machine learning algorithms, and network analysis. In spite of the promising results these methods have produced in detecting irregularities in election data, real-world applications remain challenging, particularly when dealing with complex and evolving forms of fraud such as election anomaly detection. Although the Benford and Hartigan dip test has its strengths, it should be noted that they are not foolproof and cannot definitively prove or disprove fraud, anomalies or irregularities. It serves as an initial screening tool, highlighting areas that may require further investigation or more rigorous analysis. Therefore, continued research and innovation in this area is key for the development of more effective and accurate methods for detecting election anomalies and promoting transparency and accountability in democratic societies.

*Funding statement*

This research did not receive any specific grant from funding agencies in the public, commercial, or not-for-profit sectors.

*Additional information*

No additional information is available for this paper.

## CRediT authorship contribution statement

Edmund Fosu Agyemang: Conceived and designed the experiments; Performed the experiments; Analyzed and interpreted the data; Wrote the paper.

Ezekiel Nii Noye Nortey: Conceived and designed the experiments; Contributed reagents, materials, analysis tools or data; Wrote the paper.

Richard Minkah: Performed the experiments; Analyzed and interpreted the data; Wrote the paper.

Kwame Asah-Asante: Conceived and designed the experiments; Contributed reagents, materials, analysis tools or data; Wrote the paper.

## Declaration of Competing Interest

The authors declare that they have no known competing financial interests or personal relationships that could have appeared to influence the work reported in this paper.

## Data Availability

The data used to support the findings of this study are available from the corresponding author upon request and can also be assessed from the website of the Electoral Commission of Ghana at https://ec.gov.gh/.

## References

[1] Clarke Ellis (1992).

[2] New Patriotic Party (Ghana) (1993).

[3] Nugent P. (1995).

[4] Nugent Paul (2001). Winners, losers and also rans: money, moral authority and voting patterns in the Ghana 2000 election. Afr. Aff..

[5] Gyimah-Boadi Emmanuel (2009). Another step forward for Ghana. J. Democr..

[6] Asante William, Asare Bossman E. (2017). Selected Issues in Ghana's Democracy.

[7] Adams Samuel, Asante William (2019). Biometric election technology, voter experience and turnout in Ghana. J. Afr. Elect..

[8] Agyemang Edmund Fosu, Nortey Ezekiel N.N., Minkah Richard, Asah-Asante Kwame (2023). The unfolding mystery of the numbers: first and second digits based comparative tests and its application to Ghana's elections. Model Assist. Stat. Appl..

[9] Nortey Ezekiel N.N., Agyemang Edmund F., Minkah Richard, Asah-Asante Kwame (2022). Bayesian estimation of presidential elections in Ghana: a validation approach. Afr. J. Appl. Stat..

[10] Mueller Susanne D. (2011). Dying to win: elections, political violence, and institutional decay in Kenya. J. Contemp. Afr. Stud..

[11] Breunig Christian, Goerres Achim (2011). Searching for electoral irregularities in an established democracy: applying Benford's law tests to Bundestag elections in unified Germany. Elect. Stud..

[12] Klimek Peter, Yegorov Yuri, Hanel Rudolf, Thurner Stefan (2012). Statistical detection of systematic election irregularities. Proc. Natl. Acad. Sci..

[13] Tunmibi Sunday, Olatokun Wole (2021). Application of digits based test to analyse presidential election data in Nigeria. Commonw. Comp. Polit..

[14] Ketchley Neil (2021). Fraud in the 2018 Egyptian presidential election?. Mediterr. Polit..

[15] Weidmann Nils B., Callen Michael (2013). Violence and election fraud: evidence from Afghanistan. Br. J. Polit. Sci..

[16] Bader Max, Van Ham Carolien (2015). What explains regional variation in election fraud? Evidence from Russia: a research note. Post-Sov. Aff..

[17] Mebane Walter R. (2006).

[18] Kalinin Kirill, Mebane Walter R. (2017).

[19] Mebane Walter R. (2010). Fraud in the 2009 presidential election in Iran?. Chance.

[20] Roukema Boudewijn F. (2014). A first-digit anomaly in the 2009 Iranian presidential election. J. Appl. Stat..

[21] Cole Matthew A., Maddison David J., Zhang Liyun (2020). Testing the emission reduction claims of cdm projects using the Benford's law. Clim. Change.

[22] Burkell Jacquelyn, Regan Priscilla M. (2019). Voter preferences, voter manipulation, voter analytics: policy options for less surveillance and more autonomy. Int. Policy Rev..

[23] Paulo Norbert, Bublitz Christoph (2019). Pow (d) er to the people? Voter manipulation, legitimacy, and the relevance of moral psychology for democratic theory. Neuroethics.

[24] Mansfield-Devine Steve (2018). Hacking democracy: abusing the Internet for political gain. Netw. Secur..

[25] Daniels Gilda R. (2020).

[26] Manheim Lisa Marshall, Porter Elizabeth G. (2019). The elephant in the room: intentional voter suppression. Supreme Court Rev..

[27] Pitzer Kyle, Gunn Mcclendon Gena, Sherraden Michael (2021). Voting infrastructure and process: another form of voter suppression?. Soc. Serv. Rev..

[28] Lacasa Lucas, Fernández-Gracia Juan (2019). Election forensics: quantitative methods for electoral fraud detection. Forensic Sci. Int..

[29] Zhang Mali, Alvarez R. Michael, Levin Ines (2019). Election forensics: using machine learning and synthetic data for possible election anomaly detection. PLoS ONE.

[30] Wei Yaxing, Liang Liang, Zhou Bo, Feng Xinsong (2021). 2021 13th International Conference on Communication Software and Networks (ICCSN).

[31] Daxecker Ursula E. (2012). The cost of exposing cheating: international election monitoring, fraud, and post-election violence in Africa. J. Peace Res..

[32] Mebane Walter R. (2013). APSA 2013 Annual Meeting Paper, American Political Science Association 2013 Annual Meeting.

[33] Somerville Keith (2009). British media coverage of the post-election violence in Kenya, 2007–08. J. East. Afr. Stud..

[34] Gilbreath Dustin, Balasanyan Sona (2017). Elections and election fraud in Georgia and Armenia. Caucasus Surv..

[35] Asma Hussein (2019).

[36] Cerasa Andrea (2022). Testing for Benford's law in very small samples: simulation study and a new test proposal. PLoS ONE.

[37] Kossovsky Alex Ely (2021). On the mistaken use of the chi-square test in Benford's law. Stats.

[38] Deckert Joseph, Myagkov Mikhail, Ordeshook Peter C. (2011). Benford's law and the detection of election fraud. Polit. Anal..

[39] Siffer Alban, Fouque Pierre-Alain, Termier Alexandre, Largouët Christine (2018). Proceedings of the 24th Acm Sigkdd International Conference on Knowledge Discovery & Data Mining.

[40] Hartigan P.M. (1985). The dip test of unimodality. Ann. Stat..

[41] Freeman Jonathan B., Dale Rick (2013). Assessing bimodality to detect the presence of a dual cognitive process. Behav. Res. Methods.

[42] Kang Young-Jin, Noh Yoojeong (2019). Development of Hartman's dip statistic with bimodality coefficient to assess multimodality of distributions. Math. Probl. Eng..

[43] Shanaev Savva, Shuraeva Arina, Ghimire Binam (2020).

[44] Mebane Walter R. (2006). Summer Meeting of the Political Methodology Society, UC-Davis, July.

[45] Mebane Walter R. (2011). Comment on “Benford's law and the detection of election fraud”. Polit. Anal..

[46] Nye John, Moul Charles (2007). The political economy of numbers: on the application of Benford's law to international macroeconomic statistics. B.E. J. Macroecon..

[47] Nigrini Mark J., Miller Steven J. (2009). Data diagnostics using second-order tests of Benford's law. Audit. J. Pract. Theory.

[48] Nigrini Mark J. (2012).

[49] Morzy Mikołaj, Kajdanowicz Tomasz, Szymański Bolesław K. (2016). Benford's distribution in complex networks. Sci. Rep..

[50] Leemis Lawrence M., Schmeiser Bruce W., Evans Diane L. (2000). Survival distributions satisfying Benford's law. Am. Stat..

[51] Levin Inés, Cohn Gabe, Ordeshook Peter C., Alvarez R. Michael (2009). EVT/WOTE.

[52] Pericchi Luis, Torres David (2011). Quick anomaly detection by the Newcomb—Benford law, with applications to electoral processes data from the USA, Puerto Rico and Venezuela. Stat. Sci..

[53] Hicken Allen, Mebane Walter R. (2015). U Michigan wp.

[54] Ciofalo Michele (2009). Dipartamento di Ingenieria Nucleare.

[55] Janvresse Élise, De la Rue Thierry (2004). From uniform distributions to Benford's law. J. Appl. Probab..

[56] Koch Christoffer, Okamura Ken (2020). Benford's law and Covid-19 reporting. Econ. Lett..

[57] Tam Cho Wendy K., Gaines Brian J. (2007). Breaking the (Benford) law: statistical fraud detection in campaign finance. Am. Stat..

[58] Mebane W. (2020).

[59] Myagkov Mikhail, Ordeshook Peter C., Shakin Dimitri (2009). The Forensics of Election Fraud: Russia and Ukraine.

